# Design and Analysis of English Intelligent Translation System Based on Internet of Things and Big Data Model

**DOI:** 10.1155/2022/6788813

**Published:** 2022-05-19

**Authors:** Li Lei, Hao Wang

**Affiliations:** ^1^School of General Education, Hunan University of Information Technology, Hunan Changsha 410151, China; ^2^School of Foreign Language, Changsha Normal University, Hunan Changsha 410100, China

## Abstract

Today, we have entered an era of big data. Under the background of global economization, communication in all walks of life is becoming more and more frequent and cross-language communication is inevitable. Cross-language communication is difficult for many people. The online translation system can greatly reduce the communication barriers between people of different languages. As an efficient tool, the translation system can realize the translation of different languages under the conditions of retaining the original semantics equivalent conversion. The article adopts the Internet of Things technology and big data model to build an English intelligent translation system, which can realize intelligent translation between multiple languages and English. The research results of the article show the following: (1) For samples with high semantic feature values, the correlation coefficient and similarity coefficient will be higher. Therefore, it can be concluded that for different semantics, the similarity is generally positively correlated with its feature value and correlation coefficient. The translation speed of the system proposed in the article is the fastest among the three translation systems. When the number of sentences is 10,000, the translation speed of the translation system proposed in the article is 5.89 seconds, the translation speed of the network multilingual translation system is 6.74 seconds, and the translation speed of the traditional translation system is 10.53 seconds. (2) The translation accuracy of the big data intelligent translation model proposed in the article is the highest among the three models. The translation accuracy of simple sentences can reach 99%. The translation accuracy of general sentences is 98%, and the translation accuracy of complex sentences is 95%. The BLEU value of the method in this paper is basically the same as that of the RNN cyclic neural network translation model. When translating general sentences, the BLEU value of the method in this paper is slightly higher than that of the RNN cyclic neural network translation model; especially when translating complex sentences by machine, the BLEU value of the method in this paper is far higher than that of the RNN translation model. (3) The average response time will increase with the increase in the number of tests, and the success rate generally remains above 98%, close to 100%, indicating that the response time of the system operation is normal. The number of designed test cases for the data processing module is 90, the number of executed test cases is 90, and the execution rate can reach 100%. Normal operation means that in the process of operation, no fault occurs. In the system load test, the load of serial number 1 is normal, the average delay is 38 seconds, the average delay of serial number 2 is 48 seconds, the average delay of serial number 3 is 59 seconds, the average delay of serial number 4 is 62 seconds, and the average delay of serial number 5 is 47 seconds. The delay of data packets under all kinds of loads can meet the standard requirements.

## 1. Introduction

In order to promote the development of the global economy, communication between all walks of life in the country is inevitable. As the carrier of communication between people, the free switching and transmission of languages in different countries is particularly important. Under the premise of retaining the original meaning of the sentence, it is very important to create an intelligent English translation system. Most translation systems can achieve normal communication in different languages, but they ignore the grammatical problems in the English translation process. The translation accuracy of the translation system can improve the quality of the English translation system and can also greatly reduce the communication barriers between different language groups. Based on the Internet of Things and big data model technology, the article designs an intelligent English translation system, which can not only realize the equivalent switching between multiple languages and English but also greatly improve the translation accuracy without affecting the original semantics. Literature [1] introduces CITAC technology for the design of intelligent full-text Chinese-English translators, providing an alternative, nontraditional approach to translate machine translation concepts into creation and reality. Literature [2] introduces the design motivation and overall architecture and describes the design concept and processing algorithm of its translation mechanism. Literature [3] puts forward relevant suggestions on the basis of analyzing the current situation of translation system development. Literature [4] focuses on the Chinese-English machine translation model based on deep neural network. Literature [5] uses a combinatorial technique to advance resource-limited implementations, introducing different types of word alignment techniques in English-Hindi translation systems. Literature [6] emphasizes word alignment of English language pairs, which defines the process of establishing better translation relationships between words in parallel or bilingual corpora. Literature [7] proposed an intelligent design method of the English automatic translation system based on phrase translation combination. Reference [8] proposes an implementation plan and related strategies for bidirectional automatic translation between English and Chinese in response to the research and development needs of Sino-Japanese international cooperation projects. Literature [9] proposed the problems existing in the design of the current translation system and the problems that should be paid attention to in the future research work. Literature [10] proposed a language analysis research study of the English translation system based on fuzzy algorithm. Literature [11] introduced an interactive intelligent tutoring system, emphasizing the feasibility of integrating these functions into a common platform. Literature [12] improved the traditional machine learning algorithm and proposed an improved model combining statistical language, factor analysis, and support vector machine. Literature [13] introduced the design of an online hybrid machine translation system. Reference [14] uses the machine learning algorithm as the system algorithm and combines the CA-IAFSA algorithm to construct an artificial intelligence-based English intelligent system. Literature [15] analyzed the shortcomings of traditional English intelligent translation and realized the optimal design of the human interface system of English intelligent translation.

## 2. Translation System Design of the Big Data Model

### 2.1. System Process Design

All the functional realization processes of the English online intelligent translation system are completed in the client and server of the system. System management, user management, use of thesaurus based on multilingual interaction, multilingual interactive English translation assistance, English translation management, and other functions are all implemented by the system client, database update based on multilingual interaction, knowledge file storage, and system maintenance, etc. The functions are implemented by the system server. It can be seen that most of the main functions of the system are completed by the server and the client is the part of the online translation assistant that interacts with the user.

### 2.2. System Design Route

The English intelligent translation system designed in this article is based on the Internet of Things technology and big data model. It preprocesses the English database and the Chinese database and can realize the free switching between multiple languages and English. The precondition of ensuring the original semantics in the following performs the equivalent conversion between different languages and English. The four different modules of the translation model have different functions. The translation model is the most direct interaction part between the system and the user. The model can intelligently judge the grammatical structure and part-of-speech features of the sentences to be translated. Through this module, the system can accept the original translation submitted by the customer. After the translation is successful, the system will automatically detect the pass rate of the translation and send it to the customer after reaching the pass rate. The technical route itinerary is shown in Figure 1.

## 3. Design of the English Intelligent Translation System

### 3.1. Algorithm Design

The realization of the English automatic translation system mainly adopts the organic combination of machine translation and semantic feature analysis. Assuming that the English automatic translation system is semantically distributed into five-tuples, namely, *O*={*C*, *H*^*c*^, *R*, *I*, *A*}, then the automatic translation system is vaguely mapped to [16]

(1) $$\begin{array}{c} \theta :S⟶S\times \left[-0.5,0.5\right],\\ \theta \left(S_{i}\right)=\left(S_{i},0\right),S_{i}\in S. \end{array}$$

Suppose the English automatic translation system phrase distribution structure model, as follows [17]:

(2) $$\begin{array}{c} O=\langle C,I,H^{c},R,A\rangle \\ O^{\prime }=\langle C^{\prime },I^{\prime },H^{c},R^{\prime },A^{\prime }\rangle . \end{array}$$

The system parameter and correlation parameter are set as [18]

(3) $$\begin{array}{c} \Delta :\left[0,T\right]⟶S\times \left[-0.5,0.5\right], \end{array}$$

which is defined as

(4) $$\begin{array}{c} \Delta \left(\beta \right)=\left\{\begin{array}{cc} s_{k}, & k=\text{round}\left(\beta \right),\\ a_{k}=\beta -k, & a_{k}\in \left[-0.5,0.5\right], \end{array}\right) \end{array}$$

where *β* represents the language evaluation set *S* obtained by a certain set method, *T* represents the number of elements contained in the language evaluation set, and *roun*  *d* represents the rounding operator.

The parameters of the system binary semantic fusion feature are set as

(5) $$\begin{array}{c} \left(\bar{s},\bar{a}\right)=\Delta \left(\frac{\sum_{j=1}^{n}\beta_{{}_{j}}\beta_{j}^{\prime }}{\sum_{j}^{n}↑\beta_{j}^{\prime }}\right), \end{array}$$

where

(6) $$\begin{array}{c} \sum_{j=1}^{n}\omega_{j}=1,\bar{s}\in S,\bar{a}\in \left[-0.5,0.5\right]. \end{array}$$

Among them, (*s*_*k*_, *a*_*k*_) represents binary semantic information, *s*_*k*_ represents the *K*-th element in *S*, and *a*_*k*_ represents the sign transition value.

### 3.2. Design of Translation Algorithm

Setting any Chinese matrix *f* and English sentence *e*, then the probability of *e* being machine-translated into *f* is *P*(*e|f*); then, the problem of machine translation of *f* into *e* can be seen as

(7) $$\begin{array}{c} \hat{e}=\arg\max P\left(e|f\right). \end{array}$$

If the lengths of English string *e* and Chinese string are 1 and *m*, there are

(8) $$\begin{array}{c} f=f_{1}^{m}=f_{1},f_{2}L,\ldots ,f_{m}. \end{array}$$

Alignment *a* can describe the position of words in Chinese sentences corresponding to words in English sentences through the existence of position information of each value. It is represented as

(9) $$\begin{array}{c} a=a_{1}^{m}=a_{1},a_{2}\ldots ,a_{m}, \end{array}$$

where

(10) $$\begin{array}{c} p\left(f,A|e\right)=p\left(m|e\right)\prod_{j=1}^{m}\left(a_{j}|a_{1}^{j-1},f_{1}^{j-1},m,e\right)\cdot p\left(f_{j}|a_{1}^{j},f_{1}^{j-1},m,e\right). \end{array}$$

The prerequisites are set up as

(11) $$\begin{array}{c} p\left(a_{j}|a_{1}^{j-1},f_{1}^{j-1},m,e\right)=\frac{1}{l+1}. \end{array}$$

The English machine translation model is set as [19]

(12) $$\begin{array}{c} h\left(p,\lambda \right)=\frac{s}{{\left(l+1\right)}^{m}}\sum_{al=0}^{l}L\sum_{a_{m}=0}^{l}\prod_{j=1}^{m}t\left(f_{j}|\alpha_{\theta }\right)-\sum_{\theta }\lambda_{\theta }\left(\sum_{l}t\left(f|e\right)-1\right). \end{array}$$

The improved parameter values are obtained by the maximum likelihood prediction method:

(13) $$\begin{array}{c} \hat{\theta }=\arg\max\prod_{s=1}^{s}p_{\theta }\left(f_{s}|e_{s}\right)\\ \hat{\gamma }=\arg\max\prod_{s=1}^{s}p\gamma \left(e_{s}\right). \end{array}$$

Then, the formula is obtained as [20]

(14) $$\begin{array}{c} {\hat{e}}_{1}^{l}=\arg\max\left\{p_{\hat{\gamma }}\left(e_{1}^{l}\right)\cdot P_{\hat{\theta }}\left(f_{1}^{J}|e_{1}^{l}\right)\right\}. \end{array}$$

The framework for obtaining extended statistical machine translation is [21]

(15) $$\begin{array}{c} {\hat{e}}_{1}^{l}=\arg\max\left\{P_{\hat{\gamma }}\left(e_{1}^{l}\right)\cdot P_{\hat{\theta }}\left(e_{1}^{J}|f_{1}^{l}\right)\right\}. \end{array}$$

### 3.3. English Signal Processing

The digital filter is used to realize the accent processing of the speech signal, and the accent detection system is perfected. The calculation formula of the emphasis processing signal *y*(*n*) is

(16) $$\begin{array}{c} y\left(n\right)=T\left[x\left(n\right)\right]=ax\left(n\right)+b. \end{array}$$

The speech signal is divided into *t* frame as

(17) $$\begin{array}{c} z\left(n\right)=\frac{1}{t}y\left(n\right). \end{array}$$

The voice signal is windowed as

(18) $$\begin{array}{c} \omega \left(n\right)=\omega \left(n\right)\times z\left(n\right). \end{array}$$

The signal profile is computed from discrete sample values as

(19) $$\begin{array}{c} X\left[K\right]=\sum_{n=0}^{N-1}x\left[n\right]e^{-j\left(2\pi /N\right)nk},k=0,1,2,\ldots ,N. \end{array}$$

A discrete speech sequence is converted to a *Mel*-frequency scale as

(20) $$\begin{array}{c} Mel\left(f\right)=2579\mathrm{lg}\left(1+\frac{f}{700}\right). \end{array}$$

## 4. Simulation Experiments

### 4.1. Experimental Data

In order to test the performance of the article translation system, 10 different translation samples were selected in the experiment for experimental test analysis and the semantic features, correlation coefficient, and similarity coefficient of different samples were recorded. In the experiment, the number of English semantic translation evaluation sets is 1024 instance sets and the number of iterations is 200. The fuzzy decision attributes of the English semantic translation accuracy evaluation are shown in Table 1 and Figure 2.

According to the experimental data in Table 1, we can conclude that the samples with high semantic feature values have higher correlation coefficients and similarity coefficients. Therefore, it can be concluded that for different semantics, the similarity is generally presented with its feature values and correlation coefficients with positive correlation features. English grammar is more complex, and the English translation sentence patterns set in the experiment are simple declarative sentences, general interrogative sentences, coordinating compound sentences, subordinate compound sentences, and special usage sentences to test the translation speed of the article translation system and the other two translation systems test the translation speed of different languages. The specific experiments are shown in Table 2 and Figure 3.

According to the experimental data in Table 2, we can conclude that the translation speed of the system proposed in the article is the fastest among the three translation systems. When the number of sentences is 10,000, the translation speed of the translation system proposed in the article is 5.89. The translation speed of the network multilingual translation system is 6.74 seconds, and the translation speed of the traditional translation system is 10.53 seconds. The experimental data also show that the performance of the intelligent translation system proposed in the article is always optimal and the translation speed is always the fastest regardless of the type of sentence.

### 4.2. Comparative Experiment

In order to monitor the performance of the English translation system based on the Internet of Things and big data model, the experimental corpus comes from multiple pairs of the Chinese-English parallel corpus provided by a company. The experiment divides the corpus into three test sets: simple sentences, general sentences, and complex sentences. According to the sentence length, the experiment will test the performance of the model proposed in the article with the RNN cyclic neural network translation model and the LSTM neural network translation model and observe the translation results of the three models. The test set classification is shown in Table 3, and the detection results are shown in Table 4 and Figure 4.

According to the experimental data in Table 4, we can conclude that the translation accuracy rate of the big data intelligent translation model proposed in the article is the highest among the three models and the translation accuracy rate for simple sentences can reach 99%. The translation accuracy of general sentences is 98%, and the translation accuracy of complex sentences is 95%. Among them, the translation accuracy of the LSTM neural network translation model is the lowest among the three models. The translation accuracy of simple sentences is 85%, the translation accuracy of general sentences is 88%, and the translation accuracy of complex sentences is 85%. The accuracy of the RNN translation model is in-between 82%. In order to make the experimental data more convincing, the experiment also recorded the BLEU value of the test set, and the specific data are shown in Table 5 and Figure 5. Among them, the BLEU value is an automatic evaluation method for machine translation. The higher the value, the better the quality of machine translation.

According to the BLEU curves of different models, we can conclude that the BLEU values of the method in this paper and the RNN cyclic neural network translation model are basically the same. When translating general sentences, the BLEU value of the method in this paper is slightly higher than that of the RNN cyclic neural network translation model. Especially in machine translation of complex sentences, the BLEU value of our method is much higher than that of the RNN translation model. Therefore, it shows that the advantage of this method is the machine translation of complex sentences, in which there are a large number of topmost noun phrases. The purpose is to eliminate some structural ambiguities and improve the accuracy of English machine translation.

### 4.3. System Testing

System testing is to test whether the system can work normally under a certain load [25]. The performance test of the English intelligent translation system studied in this article is mainly tested from three indicators: page response time, system operation stability, and system load test. In the experiment, the data processing module, the translation information processing module, and the communication processing module of the translation system are tested. The data processing module is to organize the content to be translated, the translation information processing module is the process of English translation, and the communication processing module is the detection process. Whether the translation result is qualified, the method of page response test is to observe the response time and operation stability of the system by continuously increasing the number of tests. The specific experimental conditions are as follows.

#### 4.3.1. Page Response Time Test

According to the data in Figure 6 and Table 6, we can conclude that the data processing module has the shortest response time, the number of tests is 120, and the average response time is 1.1 seconds. Under the experimental background of 120 tests, the average response time of the translation information processing module can reach 1.7 seconds; the experimental results of the communication processing module are between the data processing module and the translation information processing module. When the number of tests is 120, the average response time is 1.9 seconds. The average response time will increase with the increase in the number of tests, and the success rate generally remains above 98%, close to 100%, indicating that the response time of the system operation is normal.

#### 4.3.2. System Operation Stability Test

According to the data in Figure 7 and Table 7, we can conclude that the number of designed test cases of the data processing module is 90, the number of executed test cases is 90, the execution rate can reach up to 100%, and the execution rates of the translation information processing module and the communication processing module are maintained at more than 99%, close to 100%, indicating that the system can operate normally and no fault occurs during the operation.

#### 4.3.3. System Load Test

According to the experimental data in Table 8 and Figure 8, we can conclude that the load of serial number 1 is normal, the average delay is 38 seconds, the average delay of serial number 2 is 48 seconds, the average delay of serial number 3 is 59 seconds, the average delay of serial number 4 is 62 seconds, and the average delay of serial number 5 is 47 seconds, and the delay of data packets can meet the standard requirements under various loads. Therefore, it can be concluded that the developed network management security architecture can play a good role in protection without interfering with the normal operation of the computer network.

## 5. Conclusion

In the era of “Internet of Things +” strategy and big data, machine intelligent translation technology has been continuously improved, and with the help of core functions, translation efficiency and accuracy have been effectively improved. The English intelligent translation system designed in this article performs matching and feature extraction on the modules in the English semantic analysis process, which greatly solves the problems of long translation time and a low pronunciation success rate of other translation systems, and the translation success rate can reach more than 98%. However, there are still some shortcomings in the system. The scale of training data and the number of training times of the system are not enough. Due to the limitation of hardware conditions, in the future research work, large-scale data should be used, the number of training times should be increased, the memory capacity of the model should be increased, and the interpretability of the translation process should be enhanced.

## Figures and Tables

**Figure 1:** Technical route of the translation system.

**Figure 2:** Statistics of measurement results.

**Figure 3:** Statistical chart of translation results.

**Figure 4:** Test set translation accuracy comparison chart.

**Figure 5:** Test set BLEU curve.

**Figure 6:** Average response time curve.

**Figure 7:** Execution test case statistics.

**Figure 8:** Load test statistics.

**Table 1:** The fuzzy decision attribute table for the accuracy evaluation of English semantic translation.

Statistics object	Semantic features [22]	Correlation coefficient [23]	Similarity coefficient [24]
Sample 1	0.567	0.567	0.654
Sample 2	0.433	0.221	0.552
Sample 3	0.588	0.377	0.894
Sample 4	0.434	0.545	0.442
Sample 5	0.466	0.678	0.499
Sample 6	0.553	0.323	0.545
Sample 7	0.865	0.747	0.553
Sample 8	0.325	0.433	0.488
Sample 9	0.678	0.568	0.543
Sample 10	0.444	0.544	0.745
Full sample	0.324	0.577	0.686

**Table 2:** The translation results of the article system for different languages.

Number of sentences	Article translation system	Network multilingual translation system	Traditional translation system
1000	2.83	5.24	6.93
2000	3.04	5.51	7.04
3000	3.24	5.58	7.68
4000	3.68	5.65	7.65
5000	4.18	5.72	8.13
6000	4.46	5.95	8.52
7000	4.98	2.24	8.75
8000	5.03	6.42	8.94
9000	5.42	6.61	9.23
10000	5.89	6.74	10.53

**Table 3:** Test set classification results.

Kind of sentence	Word count	Number of sentences
Simple sentence	*N* < 8	458
General sentence	8 ≤*N* < 18	334
Complex sentence	N ≥ 18	175

**Table 4:** Test set translation accuracy comparison.

Translation method	Simple sentences	General sentences	Complex sentences
The method of this paper	0.99	0.98	0.95
The RNN translation model	0.93	0.94	0.90
The LSTM neural network translation model	0.85	0.88	0.82

**Table 5:** Test set BLEU value.

Translation method	Simple sentences	General sentences	Complex sentences
The method of this paper	34.62	34.64	33.62
The RNN translation model	33.58	32.48	32.10
The LSTM neural network translation model	31.24	31.10	30.49

**Table 6:** Page response time test results.

Testing frequency	50	60	70	80	90	100	110	120
Data processing module	0.4	0.5	0.6	0.7	0.8	0.9	1.0	1.1
Translation information processing module	1.0	1.1	1.2	1.3	1.4	1.5	1.6	1.7
Communication processing module	1.2	1.3	1.4	1.5	1.6	1.7	1.8	1.9

**Table 7:** System operation stability test.

Design test cases	90.00	120.00	150.00	180.00	210.00	240.00	270.00	300.00
Data processing module	90.00	120.00	150.00	180.00	210.00	240.00	270.00	300.00
Translation information processing module	90.00	119.52	149.25	178.92	208.53	238.08	261.57	297.00
Communication processing module	89.73	119.40	149.10	178.94	208.32	237.84	267.30	298.13

**Table 8:** System load test.

Serial number	Load situation	Packet volume	Average delay
1	Normal	47130	38
2	Light	37250	48
3	Severe	5510	59
4	Severe	7350	62
5	Alternating light and heavy	15380	47

## Data Availability

The experimental data used to support the findings of this study are available from the corresponding author upon request.
